The article "Space-Distributed Traffic-Enhanced LSTM-Based Machine Learning Model for COVID-19 Incidence Forecasting" was published in 2022. Journal: Comput Intell Neurosci.

# Space-Distributed Traffic-Enhanced LSTM-Based Machine Learning Model for COVID-19 Incidence Forecasting

**DOI:** 10.1155/2022/4307708

**Published:** 2022-11-18

**Authors:** Mario Muñoz-Organero

**Affiliations:** Telematic Engineering Department, Universidad Carlos III de Madrid, Leganes 28911, Madrid, Spain

## Abstract

The COVID-19 virus continues to generate waves of infections around the world. With major areas in developing countries still lagging behind in vaccination campaigns, the risk of new variants that can cause re-infections worldwide makes the monitoring and forecasting of the evolution of the virus a high priority. Having accurate models able to forecast the incidence of the spread of the virus provides help to policymakers and health professionals in managing the scarce resources in an optimal way. In this paper, a new machine learning model is proposed to forecast the spread of the virus one-week ahead in a geographic area which combines mobility and COVID-19 incidence data. The area is divided into zones or districts according to the location of the COVID-19 measuring points. A traffic-driven mobility estimate among adjacent districts is proposed to capture the spatial spread of the virus. Traffic-driven mobility in adjacent districts will be used together with COVID-19 incidence data to feed a new deep learning LSTM-based model which will extract patterns from mobility-modulated COVID-19 incidence spatiotemporal data in order to optimize one-week ahead estimations. The model is trained and validated with open data available for the city of Madrid (Spain) for 3 different validation scenarios. A baseline model based on previous literature able to extract temporal patterns in COVID-19 incidence time series is also trained with the same dataset. The results show that the proposed model, based on the combination of traffic and COVID-19 incidence data, is able to outperform the baseline model in all the validation scenarios.

## 1. Introduction

The coronavirus disease 2019 (COVID-19) is a respiratory illness. Since the first cases reported in the Chinese province of Wuhan in December 2019, COVID-19 has caused millions of infections and deaths worldwide. The virus has caused an outbreak of viral pneumonia, which has been named coronavirus disease (COVID-19) [1]. The rapid development of vaccines for COVID-19 has helped in the mitigation of the effects of the virus in parts of the world. However, there are still regions where the number of fully vaccinated people is still very limited [2] which may help the development of new mutations of the virus and their spread to other parts of the world. Policymakers and health systems need methods and models able to anticipate the spatial and temporal spread of the virus in order to optimally handle the scarce resources available and reduce the impact of the pandemic. Several methods have been developed in order to forecast the evolution of infected and recovered cases from the COVID-19 virus [3]. In fact, several predictive methods to forecast the dynamics of the virus are being used by policymakers in different regions of the world to mitigate the effects of the spread of the virus, to implement optimal policies, and to optimize the use of healthcare resources [4].

The article "Space-Distributed Traffic-Enhanced LSTM-Based Machine Learning Model for COVID-19 Incidence Forecasting" was published in 2022. Journal: Comput Intell Neurosci.

Several methods have been proposed in order to provide accurate estimations for the spread of the COVID-19 virus. Each method has its own requirements, provides a simplification of the underlying process, and tries to provide optimal estimations using the observed information. The different types of methods and models can be grouped in families such as epidemic, simulation-based, statistical, machine learning-based, and hybrid models. Epidemic models characterize the spread of the virus in terms of variables such as the number of infected people, recoveries, deaths, and infection rates. Compartmental-based epidemic models have been largely used, dividing the population into compartments or groups, and the dynamics of the spread of the virus is captured by mathematical expressions which define the movement of individuals among compartments. Examples of compartmental models are the susceptible, infected, and recovered (SIR) model and the susceptible, exposed, infected, and recovered (SEIR) model [5]. Simulation models are based on computational tools which capture the epidemiological characteristics of the virus and the behaviour of the population using rules which try to mimic the real world. A common simulation-based example is the agent-based model [3] which considers populations as autonomous software agents that behave following some rules and have a set of social characteristics and patterns of interactions among themselves. Statistical models describe the spread of the disease in terms of stochastic variables which can be modelled using probability functions, some of which can be observed while others can be estimated. Statistical models for COVID-19 use data to fit probability distributions to stochastic variables defining the spread of the COVID-19 virus such as the time to develop symptoms and the time to require hospitalization [6]. Machine learning-based models use observed data in order to learn the underlying patterns and are able to generalize to new data. Observed COVID-19 data are therefore used to train machine learning models trying to capture the behaviour of the pandemic. Once the models are trained, they can be used to forecast new results by feeding them with new data. Several machine learning models have been used for COVID-19 forecasting including deep learning models [7]. Compared with epidemic models, machine learning models do not have to generate a simplified system in order to characterize the spread of the virus but have to observe data samples coming from different sensors and learn from them. Finally, hybrid models have tried to combine machine learning models with epidemic models, using machine learning models to estimate some parameters needed by the epidemic models [8]. Hybrid models maintain the major simplifications inside the epidemic models but are fitted to the particular scenario of application. The authors in [9] developed a hybrid model by combining the susceptible-infectious-recovered-deceased compartmental model with machine learning strategies to better fit the mathematical model's coefficients for predicting infections, recoveries, deaths, and viral reproduction numbers. The authors in [10] also proposed a hybrid model that enhanced the predictions provided by the SIR epidemic model by tracking the changes in the policies implemented at the government level, which were used to estimate the time-varying parameters of an SIR model for forecasting the number of new infections one to four weeks in advance. The research in [11] uses a data-driven approach to incorporate the effects of the rate of vaccination on the COVID-19 epidemic curves on the basis of a modified susceptible-infected-recovered model enhanced by machine learning designs. The data-driven methodology is applied to assess the influence of the vaccines administered in Brazil on the fight against the virus. Hybrid models have also been proposed based on deep learning models. The study in [12] incorporates the epidemiological model dynamics of the SIRD model into an LSTM deep learning network, improving forecasting accuracy.

The article "Space-Distributed Traffic-Enhanced LSTM-Based Machine Learning Model for COVID-19 Incidence Forecasting" was published in 2022. Journal: Comput Intell Neurosci.

The spread of the COVID-19 virus is influenced by both space and time features [13]. The virus is propagated through people to people proximity interactions and is spread over a certain region helped by human mobility. This paper uses traffic sensed data in order to measure the mobility of the people among spatial zones and proposes, implements, and validates a new machine learning model able to forecast COVID-19 infections based on the use of recurrent neural network (RNN) implementing long short-term memory (LSTM) cells to extract patterns over both COVID-19 incidence and traffic data. The model is able to extract both the spatial and temporal patterns influencing the spread of the virus. The model is validated with real data for 20 months from the city of Madrid (Spain). The major contributions of this paper are as follows:

- Using a new deep learning model that combines both traffic and COVID-19 incidence data to optimize one-week ahead COVID-19 forecasting.
- Using traffic data to estimate mobility among adjacent zones (districts).
- Enhancing the accuracy of single zone models by combining the temporal patterns in adjacent zones modulated by inter-zone estimated mobility.
- Validating how the proposed machine learning model is able to learn spatiotemporal patterns from sequences of incidence and traffic-based mobility estimation to forecast the evolution of the COVID-19 pandemic for each zone (district) in a region.

The paper is organized as follows.  Section 1 introduces the objective and motivation of the research carried out in this paper.  Section 2 describes the related work, focusing on machine learning models for COVID-19 forecasting and showing the need for more studies considering spatial and temporal combined information and models to analyse both COVID-19 incidence and traffic data together.  Section 3 captures the description of the datasets used to validate the results of the paper and the methods used to process the data. A new machine learning model that processes both COVID-19 incidence and traffic data together to forecast one-week ahead incidence values is presented.  Section 4 describes the results for the new model applied to the dataset in Section 3. Finally, the major conclusions are captured in Section 5.

## 2. Related Research

Shallow machine learning models have been studied and validated as effective tools to model the COVID-19 outbreak since the first months of 2020. The authors in [14] provided initial benchmarking to demonstrate the potential of machine learning for future research showing promising results for models such as multilayer perceptron (MLP) and adaptive network-based fuzzy inference system (ANFIS). The research study in [15] used regression‐based, decision tree‐based, and random forest‐based models which were trained with data coming from the first months of the COVID-19 pandemic in China, and the trained model was then validated using the data from India. The model was able to estimate the positive number of cases.

Deep learning models have also been applied to the COVID-19 incidence time series data in order to try to optimize predictions. The research in [16] proposed a deep learning approach that included a recurrent neural network (RNN) based on a long short-term memory (LSTM) model for predicting the probable numbers of COVID-19 cases one-week ahead and applied the model trained with public datasets provided by the European Centre for Disease Prevention and Control to the data from Malaysia, Morocco, and Saudi Arabia. The authors in [17] proposed forecast models comprising long short-term memory (LSTM) and bidirectional long short-term memory (Bi-LSTM) for time series prediction of confirmed cases, deaths, and recoveries in ten major countries affected due to COVID-19. The authors validated that deep learning methods were able to outperform shallow models such as support vector regression (SVR).

The article "Space-Distributed Traffic-Enhanced LSTM-Based Machine Learning Model for COVID-19 Incidence Forecasting" was published in 2022. Journal: Comput Intell Neurosci.

Several research studies have compared the performance of different machine learning models when applied to forecast the evolution of the COVID-19 incidence, recovered cases, and deaths. The study in [18] investigated the performances of deep learning methods, including the hybrid convolutional neural network-long short-term memory (LSTM-CNN), the hybrid gated recurrent unit-convolutional neural network (GRU-CNN), CNN, LSTM, and restricted Boltzmann machine (RBM), as well as baseline machine learning methods, such as logistic regression (LR) and support vector regression (SVR). The authors showed that the use of hybrid models (i.e., LSTM-CNN and GRU-CNN) improved the forecasting accuracy of COVID-19 future trends. The performance of the models was validated with data of confirmed and recovered COVID-19 cases from seven impacted countries: Brazil, France, India, Mexico, Russia, Saudi Arabia, and the US. A similar comparative study is presented in [19] which compared four deep learning models: long short-term memory (LSTM), gated recurrent unit (GRU), convolutional neural network (CNN), and multivariate convolutional neural network (MCNN). The authors found that the CNN model was able to provide robust long-term forecasting results in time series analysis due to its capability of essential features learning, distortion invariance, and temporal dependence learning.

The spread of the COVID-19 virus has both temporal influence and spatial influence. Several studies have tried to define models that incorporated spatial information to time series pattern extraction. The authors in [13] developed a model that integrated the characteristics of time, space, and influencing factors of the COVID-19 accumulative cases applied to three European countries with severe outbreaks (Germany, Italy, and Spain) in order to extract spatiotemporal features and predict the number of confirmed cases. Although the spatial data were limited to 3 non-adjacent countries with mobility restrictions, the model was able to outperform some of the previous machine learning models focused on single time series analysis. The study in [20] proposed a new deep learning model that combined a time pattern extraction based on the use of a long short-term memory (LSTM) recurrent neural network (RNN) over a preceding spatial analysis based on a convolutional neural network (CNN) applied to a sequence of COVID-19 incidence images. The model was validated with data from the 286 primary care health centres in the Community of Madrid (Madrid region, Spain) showing improved results when compared with previous models based on time pattern extraction and analysis. Graph neural networks have also been previously used for adding the spatial component to the propagation of a virus. The authors in [21] proposed a graph message passing framework to combine graph structures (e.g., geolocations) and time series features (e.g., temporal sequences) in a dynamic propagation process. The authors validated their approach using epidemic related datasets from the United States and Japan.

The article "Space-Distributed Traffic-Enhanced LSTM-Based Machine Learning Model for COVID-19 Incidence Forecasting" was published in 2022. Journal: Comput Intell Neurosci.

The spatial component in the COVID-19 virus propagation should incorporate the information related to the mobility of the people. The initial lockdowns in different parts of the world were intended to reduce the mobility of the people in order to control the spread of the virus. The authors in [22] analysed the changes in micro-mobility usage before and during the lockdown period exploiting high-resolution micro-mobility trip data collected in Zurich, Switzerland, showing that the number of trips decreased remarkably during the lockdown period. The study in [23] described the drastic changes in human behaviour using the analysis of highway volume data as a representation of personal activity and interaction. The authors in [24] proposed a method to measure the impact of COVID-19 on transportation to further guide agencies and residents to properly respond to changes in traffic patterns based on a traffic performance score (TPS) that incorporates multiple parameters for measuring network-wide traffic performance. From previous research, we can therefore conclude that COVID-19 has had major impact on traffic. We can also find previous studies showing that traffic has had a major influence on the spread of the virus. The study in [25] investigated the association between changes in traffic volume and the spread of COVID-19 in South Korea. The relationship between traffic and confirmed COVID-19 cases was analysed using single linear regression. The authors in [26] studied the associations between the spread of COVID-19 and human mobility/demographics in the two largest counties in Wisconsin. The study was able to track the movement of people and perform a study considering and differentiating business foot traffic, race and ethnicity, and age structure. Different movement patterns by different groups resulted in different propagation speeds for the virus. Other related studies have also used data from the mobility of mobile devices in order to add spatial information to estimate the spread of the COVID-19 pandemic. The authors in [27] used the cellular network traffic data to model and forecast the number of COVID-19 infections. The paper analysed cellular network connections from 973 antennas for all users in the city of Rio de Janeiro and its suburbs and developed a Markovian model that captured the mobility of individuals across the municipalities of the city. The authors showed that the proposed mobility-aware model significantly outperformed a baseline mobility-agnostic linear regression model in terms of metrics such as root mean square error (RMSE) and mean absolute error (MAE). The authors in [28] used Facebook's Social Connectedness Index and Movement Range datasets to estimate both inter-county and intra-county population movements and proposed an LSTM-based model to forecast the upcoming COVID-19 incidence that also outperformed non-mobility-aware models.

The article "Space-Distributed Traffic-Enhanced LSTM-Based Machine Learning Model for COVID-19 Incidence Forecasting" was published in 2022. Journal: Comput Intell Neurosci.

In this paper, we propose a traffic-driven mobility impact measure among adjacent zones (districts) in a city in order to provide spatial information to a new deep learning model which will use traffic mobility data to complement COVID-19 incidence time series in order to optimize one-week ahead estimations. The proposed model will combine adjacent zone mobility with COVID-19 incidence data in order to feed an LSTM-based RNN network that will extract combined mobility and COVID-19 incidence data from adjacent zones.

## 3. Materials and Methods

This section describes the datasets used in this paper to validate the results, the method proposed to estimate the mobility between adjacent zones (districts) based on traffic data, and the proposed machine learning model that combines traffic estimated mobility and COVID-19 incidence data for each zone (district) in order to optimize one-week ahead COVID-19 predictions.

### 3.1. Datasets

Two major datasets are going to be used in order to validate the results in this paper: the traffic data provided as open data for the city of Madrid by the Madrid City Hall and the COVID-19 incidence data for each zone (district) of the city of Madrid provided as open data by the Community of Madrid regional government.

Traffic data for the city of Madrid were obtained from [29]. The dataset consists of the historic data since 2013 for 4372 measuring points providing measurements every 15 minutes. The information is divided into monthly files in order to facilitate the downloading of parts of the dataset. Each measurement at each traffic sensor for a 15-minute period consists of the traffic intensity, the occupation of the road, and the average speed over an integration period for that particular traffic sensor. The traffic sensors are divided into urban sensors and highway sensors.

The article "Space-Distributed Traffic-Enhanced LSTM-Based Machine Learning Model for COVID-19 Incidence Forecasting" was published in 2022. Journal: Comput Intell Neurosci.

The location of each traffic sensor was obtained from [30]. For each sensor, the latitude and longitude of the location of the sensor are provided together with a sensor “id” which links the data with the dataset in [29]. Each sensor has also a describing name associated to the name of the street where the sensor is located and information about the district of the city where it is located. The information about whether the sensor is a highway or urban sensor is also recorded.

The locations of the traffic sensors are shown in Figure 1. Both urban and highway sensors are shown in different colours. Each sensor is located in one particular zone of the city (district). In order to show the information of a particular district, Figure 1 shows the traffic sensors for the Latina district in yellow.

The COVID-19 epidemiologic information was obtained from [31]. The dataset provides information about the confirmed cases and the cumulative incidence numbers for each health zone in the Community of Madrid region. Health zones are defined by the location of primary care health centres where PCR tests were conducted. The location for each heath zone is also provided in the dataset. Each district in the city comprises one or several health zones.  Figure 2 shows the location of the centre of each of the 143 heath zones in the city of Madrid.  Figure 2 shows each primary care centre inside the district of the city where it is located. The COVID-19 incidence information is aggregated into city districts in [32] in order to have the same spatial data distribution as the traffic information in [29].

The datasets in [31, 32] are divided into 3 major periods. The first period goes from the beginning of the pandemic in Madrid (February 25th 2020) to July 1st 2020. During this period, data were collected every day. The period captures the first weeks of the pandemic when the measuring protocols were being defined and constantly changing. During this first period, more specifically at the beginning of the period, the availability for PCR tests was not always enough to fulfil the existing need. The second period contains weekly data from July 2nd 2020 to March 29th 2022. Measuring protocols were mature and PCR tests were available to cover the need of them for all primary care health centres. In April 2022, the majority of restrictions due to the COVID-19 pandemic in Spain were lifted and so was the way in which PCR tests were performed. The datasets in [31, 32] only contain data for confirmed cases for population over 60 years of age since April 2022.

The article "Space-Distributed Traffic-Enhanced LSTM-Based Machine Learning Model for COVID-19 Incidence Forecasting" was published in 2022. Journal: Comput Intell Neurosci.

In this paper, we are going to use the period from July 2nd 2020 to March 29th 2022 because of the maturity of the data gathering process and since it is the longest homogeneous period in the dataset.

### 3.2. Traffic Model as an Estimator for Inter-District Movements

This section presents a method to estimate an inter-district mobility related indicator based on the average of the traffic intensity for the sensors at each district closest to a particular adjacent district, weighted by the proximity of the sensor to the adjacent district. The idea behind the proposed method is that the traffic that is measured closer to the border of 2 districts is more likely to cross that border (propagating the virus between the 2 districts).. The mobility impact from the traffic in district *b* to district *a* is estimated according to

(1) $$\begin{array}{c} i_{ab}=\frac{1}{\text{N}}\underset{s}{\sum }i_{s}\frac{d_{sb}}{d_{ab}}, \end{array}$$

where

- *a* and *b* represent 2 adjacent districts (district *a* and district *b*)
- *s* represents each sensor in district *b* whose closest district is *a*
- *i*_*s*_ is the traffic intensity measured at sensor *s*
- *N* is the number of sensors *s*
- *d*_*sb*_ is the distance between sensor *s* and the centre of district *b*
- *d*_*ab*_ is the distance between the centres of the districts *a* and *b*
- *i*_*ab*_ represents the average weighted traffic intensity for the traffic measured by the sensors in *b* closest to *a* weighted by a proximity measure of each sensor to zone *a*

Equation (1) compensates the different number of traffic measuring sensors in different districts by dividing the summation of the contribution of each sensor by the total number of sensors in the summation. The traffic sensors in each district are grouped according to the proximity to adjacent districts. Only sensors from *b* whose closest district is *a* will be used in equation (1). Only urban sensors are considered in equation (1) since highway sensors are more likely to capture pass by traffic (longer distance traffic) which will have very limited impact in the virus propagation between districts *a* and *b*. Equation (1) uses the traffic intensity in urban sensors in order to measure the flow of people moving and uses the relative distance from each sensor in district *b* to the centre of district divided by the distance between the centres of the districts *a* and *b* in order to estimate the relative proximity to the border between districts. Those sensors in district *b* which are closer to district *a* will pay a more significant contribution to equation (1) since they measure traffic which is more likely to cross the border betwen the 2 districts.

The article "Space-Distributed Traffic-Enhanced LSTM-Based Machine Learning Model for COVID-19 Incidence Forecasting" was published in 2022. Journal: Comput Intell Neurosci.

Figure 3 captures the average weighted traffic intensity between districts calculated using equation (1) for a particular day in the considered period. Non-adjacent districts will not be used in the model and are represented using a weighted valued of 0. As a future work, the model will be extended to estimate the interactions among non-adjacent districts based on mobility data.

### 3.3. Proposed Model for Traffic-Enhanced COVID-19 Forecasting

The proposed model is captured in Figure 4. The model uses both COVID-19 incidence and traffic data for the last 4 weeks as inputs in order to estimate the COVID-19 incidence for each district one-week ahead. The time series for the COVID-19 incidence at each district are processed together with the weighted traffic time series from adjacent districts using an LSTM-based RNN. For each district *a*, a different LSTM-based RNN is applied to the combined weighted traffic and COVID-19 incidence time series for each adjacent district in order to extract the influence over the last 4 weeks of data in adjacent districts contributing to the propagation of the virus to district *a*. The COVID-19 incidence time series data for district *a* are also fed into an LSTM-based RNN in order to extract the impact of the past values in forecasting the evolution one-week ahead. The output of each LSTM for each adjacent district will be summarized using a dense layer which will be combined as the input of a second dense layer. A final output layer will be used to generate the one-week ahead prediction for the COVID-19 incidence in district *a*.

The model in Figure 4 has been implemented using the Keras [33] library in Python. The different layers used and their interconnection for a particular set of values for its internal parameters are captured in Figure 5 (an optimization preprocessing step will be described in the next section). The input shape captures the 4-week dependency of the input data, and the output of each LSTM layer captures the number of cells used to store the memory of each LSTM layer. The model extracts the time patterns for the COVID-19 incidence data for each district using the weighted traffic for inter-district mobility estimation together with the COVID-19 incidence data and uses a final dense layer to provide a summary for each district to learn the spatial dependencies when combining adjacent districts.

### 3.4. Baseline Model for COVID-19 Incidence Forecasting

In order to compare the forecasting accuracy of the model in Figure 5, this section captures the details of a baseline model based on the pattern extraction from COVID-19 incidence time series data similar to previous models used in related studies that will be used in the result validation section. The model is presented in Figure 6 and will be applied to the same dataset described in this section (using 4 weeks of input data to estimate the COVID-19 incidence for a district one-week ahead). The model in Figure 6 uses an LSTM-based RNN to analyse the COVID-19 incidence time patterns of a single district and uses a final processing based on a dense and an output layers. Previous studies have used similar models to process COVID-19 time series. The study in [18] optimized an LSTM-based model also using 3 layers (the third layer is the output layer). The authors in [18] required 200 epochs for training the model. The authors in [19] also used a 3-layer approach for the LSTM-based model requiring 1000 epochs for training. In order to have a fair comparison, instead of using the accuracy results from [18, 19] that were obtained using different datasets, the model in Figure 6 has been implemented in Keras [33] and applied to the same dataset as the model in Figure 5.

The article "Space-Distributed Traffic-Enhanced LSTM-Based Machine Learning Model for COVID-19 Incidence Forecasting" was published in 2022. Journal: Comput Intell Neurosci.

## 4. Results and Discussion

### 4.1. Optimization for the Model Internal Parameters

The model in Figure 5 can be tuned based on its internal parameters to optimally learn from the dataset described in the previous section. Two major parameters have been used in the optimization process:

- The number of memory units in each LSTM cell.
- The number of neurons used in the dense (fully connected) layers.

In order to simplify the optimization process, all the LSTM layers for processing the input signals have been configured with the same internal configuration. The 2 dense layers have also been configured with the same number of neurons. As a future work, other configurations will be tested in order to further optimize results.

A grid search approach has been used to train the model in Figure 5 with all the different combinations for the optimization of the 2 parameters. Both the number of memory units and the neurons in the dense layers have used a range from 2 to 14 in steps of 2. The model in Figure 5 is initialized with each combination of values, and the internal weights of the model are reset before the training of the model for each combination. A 10-fold cross validation approach is used, and the mean square error (MSE) for the validation set is used in order to assess the capacity of the model to learn the patterns in the dataset. In order to speed up the training and provide a fair comparison for MSE values among different districts, a data normalization process is used so that the COVID-19 incidence time series for all the districts are normalized using a min-max scaler between 0 and 1.  Figure 7 captures the MSE values for the different optimization parameter values.

The article "Space-Distributed Traffic-Enhanced LSTM-Based Machine Learning Model for COVID-19 Incidence Forecasting" was published in 2022. Journal: Comput Intell Neurosci.

The same optimization process has been carried out for the baseline model in order to provide a fair comparison between models.  Table 1 captures the optimal values for the models when using a 10-fold cross validation schema. The number of memory units and neurons in fully connected layers is a bit higher in the baseline model (compensating the simplicity of the model with the added complexity of a higher internal dimensionality).

### 4.2. Model Validation Results

The model in Figure 5 has been trained and validated with the datasets in [29–32], and both the mean square errors (MSEs) and the mean absolute percentage errors (MAPEs) have been compared for those achieved by the baseline model in Figure 6. The COVID-19 incidence data contain weekly data from July 2nd 2020 to March 29th 2022, and a similar time interval has been selected for the traffic data. This period contains the second to the sixth COVID-19 waves in the Community of Madrid region.

Three different validation approaches have been used in order to better assess the results and their generalization:

- A 10-fold cross validation approach which randomly splits the data in the dataset into 10 different segments of data. Each data segment is used once as the validation set. Finally, the results are averaged. This validation approach makes it easier for the model to learn the internal patterns in the validation data since there are adjacent similar data samples in the training set.
- A leave one district out validation approach which uses the entire time series for all the districts except one for training and the left-out district is then used for validation. The process is then repeated for all the districts, and the average of the MSE and MAPE values is computed. This validation approach allows us to assess if time patterns learnt from different zones generalize to new zones.
- A leave one wave out validation approach which removes the data from an entire wave in the time series for training and uses the information for that wave for validation is used. This approach is used to assess if the patterns learnt from previous waves of data generalize to new waves. The information in the dataset contains data from the second to the sixth wave. The last wave was dominated by the omicron COVID-19 variant and exhibited a particular behaviour. Therefore, the information in the fifth wave has been used to implement this validation approach.

Table 2 captures the results for the 3 validation approaches. The best results in terms of MSE values for both the proposed and the baseline models are obtained for the 10-fold cross validation schema which could be expected since the data in the training and validation subsets are similar. The MAPE values give more importance to prediction errors where the incidence values are smaller. The optimal MAPE values for the proposed model are also achieved for the 10-fold cross validation schema where the results in terms of the MAPE values for the base line model are similar for the 3 validation schemas. The proposed model in Figure 5 outperforms the baseline model for all the validation approaches. Adding the traffic data to infer inter-district mobility patterns and enhancing predictions by injecting data from adjacent districts modulated by mobility data can provide more information to the model in order to optimize the predictions. For the proposed model in Figure 5, the leave one district out approach provides better results compared to the leave the fifth wave out schema (both in terms of MSE and MAPE values). This result shows that there is a better correlation between districts for the same wave of COVID-19 infections than for different waves in the same district. The baseline model provides similar results for both leave one district and one wave out validation approaches (both in terms of MSE and MAPE values), showing that traffic modulated information from adjacent districts plays an important role both when leaving one district out and when predicting the incidence for a new wave of infections.

The article "Space-Distributed Traffic-Enhanced LSTM-Based Machine Learning Model for COVID-19 Incidence Forecasting" was published in 2022. Journal: Comput Intell Neurosci.

The average improvement rates for the 3 validation schemes in terms of MSE values when using traffic information (model in Figure 5) compared with baseline model in Figure 6 for some districts are captured in Table 3. The average improvement rate for a particular district is calculated by using only the data for that district for validation for each of the 3 validation approaches and for both models in Figures 5 and 6 and computing the average according to

(2) $$\begin{array}{c} AIr_{\text{district}}=\frac{1}{3}\underset{v}{\sum }\frac{MSE_{\text{Fig}6}\left(\text{district}\right)}{MSE_{\text{Fig}5}\left(\text{district}\right)}, \end{array}$$

where

- AIr is the average improvement rate
- *v* represents each validation approach

The geographic locations for the districts with higher improvement rates in Table 3 are captured in Figure 8 (in blue). Both Madrid-Centro and Madrid-Salamanca districts are in the centre of the city with important flows of people visiting them both for work and leisure activities.

The results for the 10-fold cross validation approach for the particular district of Madrid-Salamanca are shown in Figures 9 and 10. Both models achieve good one-week ahead forecasting results, but the model in Figure 9 (implementing the proposed model in Figure 5) has better performance estimating the peak values for the second, third, and fifth waves and is able to better follow the real upcoming infections in the initial part of each wave.

The article "Space-Distributed Traffic-Enhanced LSTM-Based Machine Learning Model for COVID-19 Incidence Forecasting" was published in 2022. Journal: Comput Intell Neurosci.

The results for the leave one district out validation approach for the same district of Madrid-Salamanca are presented in Figures 11 and 12. The proposed model in Figure 5 is able to follow the curve of real cases although there is a higher error when estimating the peak values for the COVID-19 waves. The degradation of the baseline model is higher and can be observed in both the peak values and the delays in following the increase in expected cases.

The results for the leave the 5th wave out validation approach are captured in Figures 13 and 14 (for the same district in Madrid as in the previous approaches). The proposed model is able to follow the shape of the 5th wave although the peak value is estimated with a higher error. There is also a higher delay in anticipating the increase or decrease of the number of new COVID-19 cases. The results for the baseline model are visually worse, in particular for the 5th wave which is the one used in the validation set, in which the baseline model anticipates 2 peak values of infections (while there is only one in the real data).

The results in Tables 2 and 3 and in Figures 9–14 show that using the traffic data to estimate inter-district interactions and adding traffic modulated COVID-19 incidence data from adjacent districts in a city can generate better predictions compared to a similar baseline model that only uses COVID-19 incidence data for one zone at a time (as previously used in related literature such as [18, 19]). As a future work, the model in Figure 5 could be further optimized using different LSTM layers and different pattern extraction for adjacent and predicted zones.

## 5. Conclusions

This paper has proposed and validated a new deep learning LSTM-based model able to learn from both human mobility and COVID-19 incidence time series. The model processes COVID-19 geolocated information by dividing a geographical area into zones or districts and performing their independent COVID-19 detection of new cases. Traffic dada are used to estimate the degree of interaction between adjacent districts in order to modulate the influence of the current COVID-19 incidence values from adjacent districts when forecasting the number of new cases in the district of interest. The spatiotemporal COVID-19 incidence information for each adjacent district is processed together with the estimated mobility data using an LSTM layer. The output for each district is summarized by a dense (fully connected) layer, and combined patterns are extracted by processing together the information from all the adjacent districts using fully connected layers.

The article "Space-Distributed Traffic-Enhanced LSTM-Based Machine Learning Model for COVID-19 Incidence Forecasting" was published in 2022. Journal: Comput Intell Neurosci.

The proposed model has been trained with open data for the city of Madrid and has been validated using 3 different validation approaches: 10-fold cross validation, leave one district out, and leave one COVID-19 wave out. The mean square error (MSE) and the mean absolute percentage error (MAPE) values have been compared with a baseline model used in previous literature and optimized and trained for the same dataset. The proposed model has outperformed the baseline model by reducing the MSE in 4.37, 6.01, and 2.40 times correspondently. Results show that adjacent geographical zones have an influence in the spread of the virus and that the estimation of mobility between zones helps in improving the achieved accuracy.

The current model only uses mobility estimates for adjacent zones. As a future work, a new model to estimate mobility for non-adjacent zones will be studied. The current model is based on traffic mobility data. There also exist open datasets capturing pedestrian mobility and shared bike mobility. As a future work, these datasets will be used to enhance the mobility estimation model. Finally, there are other factors that influence the propagation of the virus such as the use of masks and the percentage of people vaccinated. As a future work, the model will be expanded to use vaccination and use of mask data as inputs to complement the mobility information to better estimate the propagation of the COVID-19 virus.

## Figures and Tables

**Figure 1:** Location of the traffic sensors in the city of Madrid.

**Figure 2:** Location of the primary care health centres performing PCR testing in the city of Madrid.

**Figure 3:** Average weighted traffic intensity.

**Figure 4:** Proposed traffic-enhanced machine learning model for COVID-19 incidence forecasting.

**Figure 5:** Implemented model in Keras.

**Figure 6:** LSTM-based baseline model.

**Figure 7:** MSE for the different configuration parameters.

**Figure 8:** Districts showing better results in predictions when using traffic information.

**Figure 9:** 10-fold cross validation results for the proposed model.

**Figure 10:** 10-fold cross validation results for the baseline model.

**Figure 11:** Leave one district out cross validation results for the proposed model.

**Figure 12:** Leave one district out cross validation results for the baseline model.

**Figure 13:** Leave one wave out cross validation results for the proposed model.

The article "Space-Distributed Traffic-Enhanced LSTM-Based Machine Learning Model for COVID-19 Incidence Forecasting" was published in 2022. Journal: Comput Intell Neurosci.

**Figure 14:** Leave one wave out cross validation results for the baseline model.

**Table 1:** Optimal configuration values.

Optimal values for 10-fold cross validation	Proposed model	Baseline model
Number of memory units in the LSTM cells	4	6
Number of units in the fully connected layer	8	10

**Table 2:** Validation results for the different validation approaches.

Validation scheme	MSE (proposed model)	MSE (base model)	MAPE (proposed model)	MAPE (base model)
10-fold cross validation	0.00037	0.00162	0.2515	0.6219
Leave one district out	0.00089	0.00535	0.3122	0.7041
Leave 5th wave out	0.00193	0.00464	0.3621	0.6798

**Table 3:** Average improvement rates for different districts when using traffic information.

District	Average improvement rate
Madrid-Salamanca	5.41
Madrid-Chamartín	2.45
Madrid-Centro	4.02
Madrid-Moncloa-Aravaca	2.75
Madrid-Chamberí	2.74

## Data Availability

All the data used are open access and can be obtained in the links in references [29–32].
